The article "HPV16 E7-Dependent Transformation Activates NHE1 through a PKA-RhoA-Iinduced Inhibition of p38alpha" was retracted in 2019. Reason: concerns about the images.

# HPV16 E7-Dependent Transformation Activates NHE1 through a PKA-RhoA-Iinduced Inhibition of p38alpha

**DOI:** 10.1371/journal.pone.0003529

**Published:** 2008-10-27

**Authors:** Rosa A. Cardone, Giovanni Busco, Maria R. Greco, Antonia Bellizzi, Rosita Accardi, Antonella Cafarelli, Stefania Monterisi, Pierluigi Carratù, Valeria Casavola, Angelo Paradiso, Massimo Tommasino, Stephan J. Reshkin

**Affiliations:** 1 Department of General and Environmental Physiology, University of Bari, Bari, Italy; 2 Clinical Experimental Oncology Laboratory, National Cancer Institute Giovanni Paolo II, Bari, Italy; 3 Department of Respiratory Medicine, University of Bari, Bari, Italy; 4 Infections and Cancer Biology Group, IARC-WHO, Lyon, France; University of Hong Kong, China

## Abstract

**Background:**

Neoplastic transformation originates from a large number of different genetic alterations. Despite this genetic variability, a common phenotype to transformed cells is cellular alkalinization. We have previously shown in human keratinocytes and a cell line in which transformation can be turned on and followed by the inducible expression of the E7 oncogene of human papillomavirus type 16 (HPV16), that intracellular alkalinization is an early and essential physiological event driven by the up-regulation of the Na/^+^H^+^ exchanger isoform 1 (NHE1) and is necessary for the development of other transformed phenotypes and the *in vivo* tumor formation in nude mice.

**Methodology:**

Here, we utilize these model systems to elucidate the dynamic sequence of alterations of the upstream signal transduction systems leading to the transformation-dependent activation of NHE1.

**Principal Findings:**

We observe that a down-regulation of p38 MAPK activity is a fundamental step in the ability of the oncogene to transform the cell. Further, using pharmacological agents and transient transfections with dominant interfering, constitutively active, phosphorylation negative mutants and siRNA strategy to modify specific upstream signal transduction components that link HPV16 E7 oncogenic signals to up-regulation of the NHE1, we demonstrate that the stimulation of NHE1 activity is driven by an early rise in cellular cAMP resulting in the down-stream inhibition of p38 MAPK via the PKA-dependent phosphorylation of the small G-protein, RhoA, and its subsequent inhibition.

**Conclusions:**

All together these data significantly improve our knowledge concerning the basic cellular alterations involved in oncogene-driven neoplastic transformation.

## Introduction

Neoplastic transformation is the first step of the carcinogenic process that involves the initial altered responses of the cells to normal regulatory influences and sets the stage for further alterations that result in carcinoma. A wide variety of altered phenotypes appear as a result of transformation. Hallmarks of epithelial transformation and carcinogenesis include loss of polarity, as well as uncontrolled, serum-independent and anchorage-independent proliferation and resistance to apoptosis [1]. Other fundamental hallmarks of epithelial carcinogenesis include an elevated intracellular pH (pHi) as well as their increased rate of glucose utilization over oxidative phosphorylation [2], [3]. However, our understanding of the sequence of early events mediating the initiation, development and regulation of malignant transformation is still incomplete.

The article "HPV16 E7-Dependent Transformation Activates NHE1 through a PKA-RhoA-Iinduced Inhibition of p38alpha" was retracted in 2019. Reason: concerns about the images.

One major group of cellular signal transduction components implicated in carcinogenesis are the mitogen-activated protein kinases (MAPKs). Altered expression/activity of each of the MAPKs such as ERK (extracellular signal-regulated kinase), JNK (Jun N-terminal kinase) and p38 has been linked to tumor progression in a wide variety of cellular contexts [4]–[6]. In particular, mounting evidence indicates a negative role for the p38alpha MAP Kinase in chemical-[7] and oncogene-[8] induced tumor formation and proliferation [9], in tumor cell directed cell polarity [10]–[12] and in malignant invasion [11], [12]. Conversely, a positive role of p38 has been shown in tumor suppression and delay of tumorigenesis [13], [14], in induction of apoptosis [15], [13], [16], in a specific tumor-suppressing defense mechanism of normal non transformed cells known as oncogene induction of senescence, [17], in dormancy [18], [19] and in the increased cell viability and enhanced growth of HPV-induced recurrent respiratory papillomatosis [20]. The importance of p38 as tumor suppressor is highlighted by recent attempts to identify cancer-associated mutations in protein kinase genes, which revealed that several components of the p38 pathway, including p38alpha, are mutated in human tumors [17]. Further, p38 is activated in cancer cells during paclitaxel-driven [21], cisplatin-driven [22] and ROS-driven [23] apoptosis. In liver cells chemically induced to form tumors, p38alpha negatively regulated tumor proliferation via a repression of the JNK-c-Jun pathway [24].

While the negative role for p38alpha in regulating carcinogenesis is well described, whether it plays a similar negative role in the initiation of neoplastic transformation and through which signaling pathways are still undetermined. In this context, important questions concern if p38alpha plays a role in the development of the initial transformed phenotype after oncogene expression, what is its pattern of involvement and what are its critical upstream and downstream components. Recent progress suggests possible candidate signal transduction pathways. As a regulator of gene expression, cell cycle progression and actin cytoskeleton organization, it is now clear that RhoA, a member of the Rho family of GTPases, plays a central role in carcinogenesis and tumor progression [25]–[27]. Recent studies indicate RhoA as a central upstream regulator of MAP kinase activity [26], [28]–[31] and specifically in breast cancer [11] and pancreatic carcinoma [32] cells. Importantly, forced expression of the E7 oncogene of HPV16 in keratinocytes has recently been shown to inhibit RhoA activity although the mechanism is still not completely clear [33].

The article "HPV16 E7-Dependent Transformation Activates NHE1 through a PKA-RhoA-Iinduced Inhibition of p38alpha" was retracted in 2019. Reason: concerns about the images.

The cAMP/PKA system has been demonstrated to be involved in both transformation/tumor progression [11], [34], [35] proliferation [35]–[37] and apoptosis [38]–[40]. This system is also involved in regulating p38 activity [11], [41]–[43] and there is evidence that direct PKA-dependent phosphorylation of RhoA at Ser 188 inhibits its activity in endothelial cells [44], in smooth muscle cells [45], in cytotoxic lymphocytes [46] and in tumor cells [11] suggesting that PKA and RhoA could regulate p38 activity through a common pathway.

The goal of the present work is to determine which signal transduction systems are involved in transformation driven by a relevant oncogene. That little is known about the modifications occuring in the regulatory pathways during malignant transformation has been due, in part, to the lack of experimental models in which the transformation of normal cells by a relevant oncogene can be finely controlled and followed [17]. Since the human papilloma viruses, especially HPV16, are the prime cause of the majority of virus-associated carcinomas and the E7 and E6 proteins are the viral proteins responsible for malignant transformation [47], we chose the E7 oncogene of HPV16 to create an experimental cell model useful for the investigation of the alterations in signal transduction mechanisms underlying the initial phases of the shift from the normal to transformed state [48]. This cell model (2BN11 cells) consists of normal NIH-3T3 fibroblasts stably transfected with the gene for the HPV16 E7 oncoprotein in a vector in which its expression is under the control of a tetracycline (tet) inducible promoter such that the level of E7 expression and, therefore, transformation can be tightly regulated. This inducible expression permits the repeated following of the time-dependent development of the events in which the same cell constitutes its own control. Using the 2BN11 model system, we previously observed that intracellular alkalinization driven by an up-regulation of the Na^+^/H^+^-exchanger (NHE1) is a very early physiological event in transformation and is essential for the development of other transformed phenotypes such as increased glycolytic metabolism, increased growth rate and both serum-independent and anchorage-independent growth [48]. Here, we report that HPV16 E7-dependent transformation mediated by NHE1 is driven by the action of a RhoA-p38alpha module gated by the PKA dependent phosphorylation of RhoA.

The article "HPV16 E7-Dependent Transformation Activates NHE1 through a PKA-RhoA-Iinduced Inhibition of p38alpha" was retracted in 2019. Reason: concerns about the images.

## Materials and Methods

### Cell culture, transfections and reagents

NIH3T3 cells were cultured in Dulbecco's modified Eagle's medium (DMEM) with 4.5 g of glucose per liter, supplemented with 10% calf serum. Normal human foreskin keratinocytes (HFKs) were isolated from neonatal foreskin as described previously [49] and were maintained in keratinocyte growth medium supplemented with bovine pituitary extract (Clonetics). Primary human keratinocytes infected with HPV16 [50] and cultured at low (HPK1a early) or high (HPK1A late) passage numbers were maintained as previously described [48]. These cells spontanously transform at high passages and high passage cells are tumorgenic in nude mice [48].

High-titer retroviral supernatants (10^6^ virus particles/ml) were generated by transient transfection of Bosc23 cells (ecotropic viruses) or Phoenix (amphotropic viruses) and used to infect the cells as described previously [48]. Cells were grown to about 80% confluence in a 10-cm-diameter dish and infected with 5 ml of the recombinant retrovirus or parental virus in the presence of 8 µg of Polybrene per ml in order to enhance infection efficacy. After 6 h infected cells were fed with complete medium and kept at 37°C with 5% CO_2_ for 48 h. The cells were then transferred to four 10-cm-diameter dishes and selected with 2.0 µg of puromycin/ml for 3 to 4 days. Selected cells were expanded and used for experiments, generally when at 80% confluence. NIH3T3 or HFK cells were infected with recombinant retrovirus (pLXSN vector, Clontech, BD, Le Pont Claix, France) expressing non-tagged HPV16 E7 proteins. In some experiments, NIH3T3 cells constitutively expressing E7 genes were generated by infection with pBabepuro vector expressing HPV16 HA-tagged E7 proteins, wild-type or mutant.

The 2BN11 cell line was created by infecting NIH3T3 cells with recombinant retrovirus expressing the HPV16 E7 gene under the control of a tetracycline repressed promoter. The tetracycline-controlled expression system consisted of regulator and response elements in a one vector system [48]. Cells were cultured in DMEM high glucose (4500 mg/l) supplemented with NaHCO_3_ (3700 mg/l), 10% (v/v) heat inactivated fetal bovine serum, L-glutamine (2 mM), Na-Pyruvate (1 mg/ml) and 1 µM tetracycline. The clones, after selection in puromycin, were selected on the basis of having low basal E7 expression in the presence of tetracycline and high inducibility as determined by Western blot and RT-PCR analysis.

The article "HPV16 E7-Dependent Transformation Activates NHE1 through a PKA-RhoA-Iinduced Inhibition of p38alpha" was retracted in 2019. Reason: concerns about the images.

Transient transfections with the various mutated cDNAs were performed with the FuGENE HD Transfection Reagent (Roche) according to the manufacturer's instructions [12]. H89, SB203580 and IBMX were purchased from Sigma whereas Forskolin was from Calbiochem (Novabiochem Corp., La Jolla, CA). The effect of these clones or pharmacological agents on E7 expression were tested in an RT-PCR assay as described below and none of them had any effect on E7 message (Figure S1)

### RNA preparation and semiquantitative RT-PCR

Total RNA was extracted from cells using the RNeasy system (Qiagen, Valencia, CA) and treated with RNAase-free Dnase (Qiagen) for 15 min at room temperature. Spectrophotometric ratios of A260 to A280 were greater than 1.8. Total RNA (500 ng) was reverse transcribed in 20 µl reaction system using Random Hexamers priming and MuLV Reverse Transcriptase (RT) with the RNA PCR Kit GeneAmp (Applied Biosystems) under conditions described by the supplier. Reverse transcription-PCRs (RT-PCRs) were carried out essentially as previously reported [12]. Quantification of HPV16 E7 expression levels was performed by comparison to the GAPDH (glyceraldehyde-3-phosphate dehydrogenase) housekeeping gene. Primer sequences were as follows: HPV16 E7 gene, 5′-ATG CAT GGA GAT ACA CCT AC-3′ (forward) and 5′-TAT GGT TTC TGA GAA CAG ATG-3′ (reverse); GAPDH gene, 5′-ACC ACA GTC CAT GCC ATC AC-3′ (forward) and 5′-TCC ACC ACC CTG TTG CTG TA-3′ (reverse). PCRs for HPV16 E7 and the GAPDH gene were performed by a touchdown protocol with the following cycling conditions: 10 min at 95°C (initial denaturation), 6 cycles of step-down PCR consisting of 45 s at 95°C (denaturation), 60 s at 58°C (annealing) – decrease 1°C each cycle until 53°C; and 120 s at 72°C (extension). Amplification of the final product was completed for 26 cycles of 45 s at 95°C, 60 s at 53°C, and 120 s at 72°C, with a final extension of 10 min at 72°C. In the negative control, RNase free water (Gibco) was used instead of template RNA. The positive control included HPV16 E7 cDNA. Amplicons were separated on 1.5% agarose gel and visualized by ethidium bromide staining.

### NHE1 activity

Intracellular pH was determined spectrofluorimetrically in cells loaded with the acetoxy-methyl ester derivative of the pH-sensitive dye 2,7-biscarboxyethyl-5(6)-carboxyfluorescein (AM-BCECF, Invitrogen). NHE1 activity was determined by measuring the rate of pHi recovery from an acid load produced with the NH4Cl prepulse technique by evaluating the derivative of the slope of the time-dependent pHi recovery (dpHi/dt) as previously described [40], [48]. The use of CO_2_/HCO_3_ free solutions minimizes the likelihood that Na^+^-dependent HCO_3_ transport was responsible for the observed pHi changes.

The article "HPV16 E7-Dependent Transformation Activates NHE1 through a PKA-RhoA-Iinduced Inhibition of p38alpha" was retracted in 2019. Reason: concerns about the images.

After each experiment trypan blue exclusion was also measured for each cover slip and when was more than 5% the experiment was not used.

### Construction of expression vectors containing RhoA mutants

Site-directed mutagenesis of RhoA to create RhoAS188A was performed by PCR overlap extension as previously described [11]. The successful construction of the mutants was confirmed by DNA sequence analysis. The cDNA were cloned into the pBabe puro expression vector containing a hemagglutinin (HA) tag.

### RhoA RNA Interference

Small interfering RNA (siRNA) duplex against RhoA (sc-29471) was obtained from Santa Cruz Biotechnology. The specificity of the silencing tecnique was verified by using a control, non targeting 20–25 nucleotide siRNA designed as a negative control (Control siRNA-A, sc-37007, Santa Cruz Biotechnology). siRNAs were used at 100 nM concentration and transfection with siRNA was performed using Lipofectamine 2000 (Invitrogen) 24 hr after plating cells. The efficiency of RhoA silencing was measured in immunofluroescence microscopy using a monoclonal anti-RhoA antibody (sc-418, Santa Cruz Biotechnology) and was found to be ∼75% after 72 hrs siRNA treatment (Fig. S2). RhoA expression levels were measured via pixel density analysis using the WCIF Image J 1.37c software (Wayne Rasband, NIH, USA). Therefore, NHE1 activity was analyzed 72 hrs post-transfection with either RhoA siRNA or control siRNA-A in the presence of tet or 24 hrs after tet removal.

### Adherent cell cAMP assay

Cells (10^4^ cells in 100 µl of media) were plated into each well of a Greiner Bio-one tissue culture grade 96-well white clear bottom microassay plate (PBI S.p.a., Italy) and incubated in 5% CO_2_ atmosphere at 37°C for 24 hr. Cells were washed once with 100 µl of DMEM serum free medium plus 100 µM IBMX and then treated with 20 µM of FSK and 1 mM of IBMX in 20 µl of reaction media at 37°C for 30 min. Levels of cytosolic cAMP were then measured with the cAMP-Glo™ assay (Promega, Italy) as per manufacturers instructions. Briefly, the medium was aspirated, 20 µl of lysis buffer and 40 µl of cAMP-Detection Solution was added and the plate was incubated with gentle rocking at room temperature for 20 min. Next, 80 µl of Kinase-Reagent were added, and luminescence was read after incubation for 10 minutes in a Fluorescence Spectophotometer Cary Eclipse VARIAN in its chemiluminescence mode where each well is read for 20 seconds. Increases in cAMP levels result in decreases in chemiluminescence.

The article "HPV16 E7-Dependent Transformation Activates NHE1 through a PKA-RhoA-Iinduced Inhibition of p38alpha" was retracted in 2019. Reason: concerns about the images.

### cAMP FRET measurements and cell imaging

For time-lapse FRET experiments, cells were cotransfected with 1.5 µg each of pcDNA3Cat-YFP and pcDNA3RII-CFP plasmids using Fugene 6 (Roche, Switzerland) for 24 hr as described [51]. Twenty-four hours after transfection, monolayers of cells were cultured an additional 3 or 24 h in the presence or absence of tetracycline and imaged on a Nikon ECLIPSE TE 2000-S equipped with a charge-coupled device camera, a controlled DeltaRAM monochromator on the excitation side and a beam splitter (Optical Insight, St. Cloud, MN) on the emission side fitted with a 505DCRX dichroic and two emission filters, D480/30 and D535/40. Excitation was at 430 nm and the dichroic mirror was a 455DRLP. Acquisition and FRET analyses were performed using the Metafluor 4.6 software (Meta Imaging 4.6; Universal Imaging, Downingtown, PA). The live imaging was done with 4×4 binning to minimize exposure time, photobleaching and registration artifacts. To study agonist-induced changes in FRET: following the recording of a baseline, cells were first continuously superfused with the phosphodiesterase inhibitor IBMX (100 µM) and then treated with a mix of IBMX (100 µM) and the adenylate cyclase activator forskolin (25 µM). The change in FRET signal due to mobilization of cAMP was detected by FRET/CFP ratiometric processing in both non stimulated and agonist-stimulated cells, in which both FRET (CFP excitation–YFP emission) and CFP (CFP excitation–CFP emission) images were first background subtracted. Cells were thresholded to discard any portions of the image with insufficient intensity to provide reasonable signal/noise. The resulting background-subtracted FRET image was divided by that of CFP image to obtain a pixel-to-pixel FRET/CFP ratio image Increasing cAMP levels result in a reduction in FRET ratio (Em YFP/Em CFP). The final FRET images were displayed in pseudocolors scaled linearly from the lowest (red) to the highest (blue) signal to show relative increase in cAMP mobilization of levels within each cell at each treatment at both 3 and 24 hrs.

### Protein extraction and Western blotting

Western Blotting was performed as described [11]. Samples were extracted in sodium dodecyl sulfate (SDS) sample buffer (6.25 mM Tris-HCl, pH 6.8, containing 10% (v/v) glycerol, 3 mM SDS, 1% (v/v) 2-mercaptoethanol and 0.75 mM of Bromophenol Blue), separated by 4–12% SDS-PAGE and blotted to Immobilon P. Analysis of phospho- and total RhoA was performed by using an antibody produced against a peptide of RhoA phosphorylated at serine 188 by PRIMM (Milan, Italy) diluted 1∶1000, against total RhoA (sc-418, Santa Cruz, CA) diluted at 1∶1000, against tubulin (T5293, Sigma) and against the HA tag (MMS-101R BabCo, diluted 1∶200). Molecular weights standards were ‘Biotinylated Protein Ladder Detection Pack’ (Cell Signaling Technology, MA).

The article "HPV16 E7-Dependent Transformation Activates NHE1 through a PKA-RhoA-Iinduced Inhibition of p38alpha" was retracted in 2019. Reason: concerns about the images.

### Phospho-Kinase Assays

For the kinase phosphorylation measurements total cellular protein was extracted in SDS-sample buffer (50 mM Tris-HCl pH 6.8, 2% SDS, 10% glycerol and 0.1% bromophenol blue) and approximately 50 µg was separated on 10% SDS-PAGE and transfered to Immobilon P, (Millipore). The relative amount of each phosphorylated kinase (ERK, JNK and p38) to its total expression was determined by Western Blotting with antibodies specific to each obtained from Cell Signaling Technology (MA, USA).

### p38 MAP kinase activity assay

To assay p38 MAP kinase activity, cells were grown to approximately 70% confluence in 10 cm plates (GIBCO) and treated as decribed in figure legends. After treatment, cells were washed with ice-cold phosphate-buffered saline (PBS) and lysed by 5 minutes at 4°C in lysis buffer (150 mM NaCl, 1 mM EDTA, 1 mM EGTA, 1% Triton X-100, 2.5 mM sodium pyrophosphate, 1 mM ß-glycerophosphate, 1 mM Na_3_VO_4_, 1 µg/ml leupeptin, 20 mM Tris, pH 7.4) plus 1 mM PMSF. The cells were scraped into Eppendorf tubes and triturated by sonification. The cell lysate was centifuged at 4°C for 10 min at 14,000 rpm and the supernatant collected. Protein levels were equalized by normalizing them to the protein levels measured before the assay.

p38 MAP kinase activity was quantified using an immune complex kinase assay kit according to the manufacturer's protocol (New England Biolabs). Briefly, cleared lysates were immunoprecipitated overnight at 4°C with p38 MAPK antibodies conjugated to agarose (New England BioLabs). Beads were washed three times with ice-cold lysis buffer and three times with kinase reaction buffer (25 mM Tris pH 7.5, 5 mM ß-Glycerolphosphate, 2 mM DTT, 0.1 mM Na_3_VO_4_, 10 mM MgCl_2_) minus ATP and ATF-2. The pellet was resuspended in 50 µl kinase reaction buffer plus 200 µM ATP and 10 µg GST-ATF-2 as substrate and incubated at 30°C for 30 minutes. The reaction was stopped by addition of 2× Laemmli buffer. The sample was run on 10% SDS-PAGE and blotted onto polyvinylidene difluoride membranes (Millipore) for immunoanalysis. The amount of ATF-2 phosphorylated by p38 was analyzed by Western blotting with a Phospho-ATF-2 (Thr71) antibody (Cell Signaling) that detects only catalytically activated ATF-2. Total p38 expression measured by immunoblotting was not found to vary under any experimental conditions.

The article "HPV16 E7-Dependent Transformation Activates NHE1 through a PKA-RhoA-Iinduced Inhibition of p38alpha" was retracted in 2019. Reason: concerns about the images.

### Analysis of RhoA serine phosphorylation state

After treatment cell monolayers were washed twice with ice-cold PBS and lysed in ice-cold RIPA (the above lysis buffer plus 0.1% SDS and 0.2% Na-deoxycholate). The cellular lysate was centrifuged at 14,000 rpm for 5 min at 4°C. Protein levels were equalized by normalizing them to the protein levels measured before the assay and the supernatent pre-cleared with protein A-agarose for 2 hrs at 4°C. Cleared lysates were immunoprecipitated overnight at 4°C with a phosphoserine antibody conjugated to agarose (SIGMA). The agarose beads were washed four times with simple RIPA buffer. The pellet was resuspended in 50 µl Laemmli buffer. The sample was run on 12% SDS-PAGE and blotted onto Immobilon P (Millipore) for immunoanalysis of the amount of RhoA immunoprecipitated by antiphosphoserine with a RhoA antibody (sc-418, Santa Cruz).

### Analysis of the activity of RhoA

RhoA activity was assessed using the RhoA-binding domain of Rhotekin in a kit supplied from Upstate Biotechnology (Lake Placid, NY). In brief, 3×10^6^ cells were plated onto 10 cm cell culture dishes and after 24 hrs treated as indicated. After the indicated time, cells were extracted with RIPA buffer (50 mM Tris, pH 7.2, 500 mM NaCl, 1% Triton X-100, 0.5% sodium deoxycholate, 1% SDS, 10 mM MgCl_2_, 0.5 µg/ml leupeptin, 0.7 µg/ml pepstatin, 4 µg/ml aprotinin, and 2 mM PMSF). After centrifugation at 14,000 g for 3 min, the extracts were incubated for 45 min at 4°C with glutathione beads coupled with GST–RBD (Rho-Binding Domain of Rhotekin) fusion protein (Upstate Biotechnology, Lake Placid, NY), and then washed three times with Tris buffer, pH 7.2, containing 1% Triton X-100, 150 mM NaCl, and 10 mM MgCl_2_. The RhoA content in these samples or in 50 µg protein of cell homogenate was determined by immunoblotting samples using anti-RhoA antibody from Santa Cruz (sc-418, Santa Cruz, CA).

### FRET assay for RhoA activity

For these experiments, endogenous RhoA activity was measured in FRET microscopy using the Raichu 1297 probe as previously described [11]. In this sensor, the Rho Binding Domain (RBD) of the RhoA effector protein, Rhotekin, is sandwiched by Venus-YFP and CFP. The binding of endogenous GTP-RhoA to RBD generates a conformational change that displaces YFP and CFP, thereby decreasing fluorescence resonance energy transfer (FRET) efficiency between the two fluorophores, while a reduction of intracellular active RhoA results in the opposite effect. The CFP channel images were divided by the YFP-FRET channel images. The activity of RhoA is monitored by measuring CFP (480 nm)/YFP(545) fluorescence emission values upon excitation of the transfected cells at 430 nm. To eliminate the distracting data from regions outside of cells, the YFP channel is used as a saturation channel. The ratio images are presented in pseudocolor mode. Ratio intensity is displayed stretched between the low and high renormalization value, according to a temperature-based lookup table with blue (cold) and red (hot) indicating respectively high and low values of RhoA activity.

The article "HPV16 E7-Dependent Transformation Activates NHE1 through a PKA-RhoA-Iinduced Inhibition of p38alpha" was retracted in 2019. Reason: concerns about the images.

Additionally, FRET was used to monitor RhoA activity due to the activity balance between endogenous guanine nucleotide exchange factors (GEFs) and GTPase-activating proteins (GAPs): cells were transfected with a plasmid with the cDNAfor Raichu-RhoA-1293, which consisted of truncated RhoA (aa 1–189), the RhoA-binding domain (RBD) of effectors, and a pair of GFP mutants, YFP and CFP. In these probes, the intramolecular binding of GTP-RhoA to the effector protein was expected to bring CFP in closer proximity to YFP, resulting in an increase in FRET from CFP to YFP.

The set up of the microscope and the filters used for FRET excitation and emission were identical to those reported for the cAMP FRET measurements. Briefly, twenty-four hours after transfection, monolayers of cells were cultured an additional 24 h in the presence or absence of tetracycline and, images from filter sets dedicated for YFP, CFP, and FRET fluors were first captured, and then three to four random regions of interest within each cell, were chosen for analysis. Sensitized FRET measurements Off-line image analysis was performed using the Metafluor 4.6 software (Meta Imaging 4.6; Universal Imaging, Downingtown, PA). Correction of FRET measurements for spectral bleedthrough and cross excitation was calculated on a pixel-by-pixel basis for the entire image by estimating net FRET (nF) as follows: nF = IFRET−(IYFP×*a*)−(ICFP×*b*), where IFRET is sensitized YFP emission (excitation 430 nm, emission 545 nm) and IYFP and ICFP are YFP emission (545 nm) upon excitation at 480 nm and CFP emission (480 nm) upon excitation at 430 nm, respectively. *a* is a norm of the percentage of CFP bleed-through, and *b* is a norm of the percentage of direct excitation of YFP at 430 nm. *a* and *b* were determined by analyzing images of cells expressing only CFP or YFP as described previously [11], and for our system a and b values corresponded to 64 and 8%, respectively. Corrected FRET ratio was calculated as ICFP/nF.

### Statistical Procedures

In the *in vitro* experiments, student's t-test was applied to analyze the statistical significance between treatments. All comparisons were performed with InStat (GraphPad Software).

The article "HPV16 E7-Dependent Transformation Activates NHE1 through a PKA-RhoA-Iinduced Inhibition of p38alpha" was retracted in 2019. Reason: concerns about the images.

## Results

Our goal was to study the signal transduction mechanisms involved in neoplastic transformation driven by a biologically relevant oncogene. The E7 oncoprotein of HPV16 is known to induce transformation both *in vitro* and *in vivo* and to fully transform immortalized rodent fibroblasts (E7/NIH3T3 cells) or human keratinocytes which are tumorigenic in nude mice [48], [50].

### HPV16 E7-induced transformation induces down-regulation of p38 but not JNK or ERK MAPKinase activity

We first determined the effect of HPV16 E7 expression on MAP Kinase activity by transducing immortalized NIH3T3 cells or human foreskin kerotinocytes (HFK), the natural host of the virus, with a recombinant retrovirus expressing non-tagged, wild-type HPV16 E7 and measuring the phosphorylation state of ERK1/2, JNK and p38 MAP kinase as described in Material and Methods. As seen in Figures 1A (NIH3T3) and 1B (HFK), E7 expression reduced the phosphorylation state of p38 MAP kinase (p38) by approximately 90% while having no significant effect on the phosphorylation level of either the ERK or JNK MAP kinases. The same results were observed in NIH3T3 cells infected with HA-tagged wild-type E7 (data not shown). Further, two different protocols were used to determine whether it is simply E7 expression or E7-dependent transformation that leads to an inhibition of p38. First, we used human primary keratinocytes (HPKIA cells) immortalized by transfection of the entire HPV16 genome and which become spontaneously transformed at high passage number and are tumorigenic in nude mice [48], [50]. As shown in Figure 1C, p38 was much less phosphorylated in the transformed (late passage) keratinocytes than in the immortalized (early passage) cells while, also here, having no significant effect on the phosphorylation levels of either the ERK1/2 or JNK MAP kinases. To further confirm this dependance of p38 dephosphorylation upon HPV-induced transformation, we then extended our study to NIH3T3 cells infected with recombinant retroviruses expressing either wild-type HPV16 E7 or transformation-deficient mutants [53], [54]. As seen in Fig. 1D, the wild-type E7 reduced p38 phosphorylation as above while the transformation negative mutants had no effect on p38 phosphorylation. Altogether, these results demonstrate that HPV16-induced transformation reduces the p38 activity through E7 without affecting either the ERK or the JNK MAP kinases and are consistent with the reported specificity of p38 in oncogenic processes.

**Figure 1:** Only HPV16 E7 expression and not other non-transforming HPV types decreases p38 MAPK phosphorylation in both NIH3T3 cells and human keratinocytes. A. Cell extracts from empty pLXSN vector NIH3T3 cells and HPV16 E7 infected cells were analyzed by Western Blot for both the phosphorylation state and total expression level of ERK, JNK and p38 MAPK. Western blot analysis was carried out using polyclonal anti-phospho-ERK1/2, anti-phospho-JNK and anti-phospho-p38 antibodies followed by polyclonal anti-total ERK1/2, total-JNK and total-p38 MAP Kinase antibodies. Tubulin expression was used as an additional loading control and 500 ng of each sample total RNA were subjected to a semi-quantitative RT-PCR for HPV16 E7 expression analysis. GAPDH: loading control, pc: positive control, nc: negative control. B. Cell extracts from empty pLXSN vector HFK cells and HPV16 E7 infected HKF cells were analyzed by Western Blot for both the phosphorylation state and total expression level of ERK, JNK and p38 MAPK as above. C. Cell extracts from early passage (p94) HPK1A cells and late passage (p396) HPK1A cells were analyzed by Western Blot for both the phosphorylation state and total expression level of ERK, JNK and p38 MAPK as above. D. NIH3T3 cells were infected with recombinant retroviruses expressing either empty vector (pBabe), wild type HPV16 E7-Ha tag (WT), or transformation-deficient HPV16 E7-Ha mutants (24, 10, 31/32), and total cell extracts were assayed in Western blot for phosphorylated and total p38 expression levels as above. All the cell lines expressed E7 as confirmed by using an Ab anti HA-tag (E7-HA). Preliminary experiments demonstrated that the HA tag does not interfer with the induction of transformation (data not shown).

The article "HPV16 E7-Dependent Transformation Activates NHE1 through a PKA-RhoA-Iinduced Inhibition of p38alpha" was retracted in 2019. Reason: concerns about the images.

### HPV16 E7-dependent down-regulation of p38 is an early event in transformation

The above experimental systems do not permit the determination of the dynamic processes occurring during transformation. To determine whether inhibition of p38 is an early event in transformation, a cell model was constructed in which the transformation of normal cells can be rapidly induced and early events subsequently monitored. NIH3T3 cells were infected with a recombinant retrovirus in which HPV16 E7 gene expression is under the control of a promoter that is negatively regulated by tetracycline, clone 2BN11 [48]. The temporal sequence of the increase in E7 message (Fig. 2A) and the change in p38 phosphorylation state (Fig. 2B) and in activity, measured as the phosphorylation of its substrate, ATF2, (Fig. 2C) was monitored after induction of E7 expression. These experiments showed that the increase in E7 mRNA and reduction of both p38 phosphorylation and activity levels started approximately 2–3 hrs after tet removal, which is in agreement with the previously observed time course for the appearance of E7 mRNA and protein [48].

The article "HPV16 E7-Dependent Transformation Activates NHE1 through a PKA-RhoA-Iinduced Inhibition of p38alpha" was retracted in 2019. Reason: concerns about the images.

**Figure 2:** Time course of changes in HPV16 E7 expression and both phosphorylation and activity of p38 MAPK in 2BN11 cells after tetracycline (tet) removal. A. The activation of HPV16 E7 transcription upon tet removal from the culture medium was determined by RT-PCR as described in in Materials and Methods. After tet removal the cells were collected at the indicated times, total RNA prepared, cDNA generated and the levels of message were determined. The levels of GAPDH were also determined in each sample as internal control. nc: negative control in which the PCR was performed in the absence of a template; pc: positive control included HPV16 E7 cDNA as template. B. Time course of HPV16 E7 expression-dependent inhibition of p38 phosphorylation, total p38 and tubulin in 2BN11 cells after tetracycline removal. C. p38 activity during HPV16 E7 expression (tet removal) was determined by exposing p38 immunoprecipitated from 1 mg of cell lysate to 10 µg GST-ATF-2 as described in methods. The amount of ATF-2 phosphorylated by p38 was analyzed by Western Blotting with an Phospho-ATF-2 (Thr71) antibody and tubulin levels in the homogenate was used as loading control.

### HPV16 E7 expression activates the cAMP pathway

As the cAMP/PKA system has been demonstrated to be involved in both transformation/tumor progression [12], [35], [55], [56] and regulation of p38 [57], we next measured the effect of E7-driven transformation on the levels of cellular cAMP at both early (3 hrs) and late (24 hrs) time points after tet removal. We started with a biochemical assay in which the bioluminescence intensity level inversely correlates with cAMP intracellular mobilization (see Materials and Methods). Cells were first treated with 100 µM of the phosphodiesterase inhibitor, IBMX, in order to observe the activity level of endogenous adenylate cyclase and then were treated with IBMX together with 20 µM of the pharmacologic adenylate cyclase activator, forskolin, to determine the dynamic range of increasing activity of the remaining non E7-stimulated enzyme. The left panel of Figure 3A shows a much greater decrease of bioluminescence after inhibition of intracellular phosphodiesterases by IBMX in the E7-transformed cells (−tet) while the subsequent decrease of bioluminescence after addition of the adenylate cyclase stimulator, forskolin, was similar in control and transformed cells. Calculation of cAMP concentration with a standard curve showed that transformation increased cellular cAMP levels (measured in the presence of IBMX), by approximately 2.5-fold at 3 hrs and 5-fold at 24 hrs without increasing total potential adenylate cyclase activity (Figure 3A right panel). Interestingly, a similar rise in cAMP was observed in late passage compared to early HPK1A cells and, further, blockage of NHE1 activity with 2 µM of its specific inhibitor, HOE642, had no effect on this E7-induced increase in cAMP in either 2BN11 or HPK1A cells (Figure S3).

The article "HPV16 E7-Dependent Transformation Activates NHE1 through a PKA-RhoA-Iinduced Inhibition of p38alpha" was retracted in 2019. Reason: concerns about the images.

**Figure 3:** HPV16 E7 expression stimulates cAMP generation in 2BN11 cells. To determine the effect of E7 expression on cAMP production, cAMP levels were measured using A. the biochemical luciferase-based Kinase-Glo System where luminescence is inversely proportional to cAMP levels (for details see Methods). Cells were cultured with or without tet for either 3 or 24 hr and then either not treated (dark bars) or treated for 30 min with either 100 µM IBMX (light bars) or 100 µM IBMX plus 20 µM FSK (stippled bars). Left panel shows levels of luminescence in the various treatments while right panel shows the calculated increase in cAMP concentration with each treatment. Error bars represent the standard error of the mean (SEM) of three independent experiments. B. Time-lapse FRET imaging in live cells transfected with a PKA-based FRET probe, in which cyan and yellow mutants of GFP have been fused to its regulatory and catalytic subunits, respectively, so that cAMP-induced dissociation between the two is detected as FRET changes. Cells were transfected with the FRET cAMP biosensor for 24 hrs and then cultured with or without tet for either 3 or 24 hr. Cells were mounted in a perfusion chamber and the FRET ratio measured during superfusion with ringer alone followed by superfusion first with 100 µM IBMX and then 100 µM IBMX plus 20 µM FSK. Cells were imaged for CFP and YFP every 20 s and the YFP/CFP emission ratios (FRET ratios) obtained. Left panel shows levels of YFP/CFP emission ratios in the various treatments while right panel shows the calculated increase in YFP/CFP emission ratios with each treatment which is relative to increases in cAMP production. Data are the mean±SEM from 32 different cells. C. Pseudocolor images representing YFP/CFP emission ratios recorded under control conditions (plus and minus tet for either 3 or 24 hrs), after exposure to 100 µM IBMX and after stimulation with IBMX (100 µM) plus FSK (20 µM). Each image was scaled according to its high and low values at each time point to show relative level of cAMP at each time point. The dynamic range was 0.9–1.3. Warmer colors correspond to lower cAMP levels.

To further verify this specific stimulation of cAMP mobilization in response to HPV16 E7 expression and visualize cAMP dynamics *in vivo*, we transfected 2BN11 cells with a PKA-based FRET construct composed of green fluorescent protein variants bound to either the PKA catalytic subunit (Cat-YFP) or the PKA regulatory II subunit (RII-CFP) and recorded FRET images with a dual-emission CCD camera. Increased levels of cAMP produce a decrease in FRET signal, measured as YFP-to-CFP emissions ratio, due to cAMP binding to the chimeric PKA reporter and the resultant separation of the catalytic and regulatory subunits. In time course experiments, when the cAMP signal was stable, cells were first treated with IBMX in order to observe the activity level of endogenous adenylate cyclase and then were perfused with IBMX together with forskolin to determine the dynamic range of increasing activity of the remaining non E7-stimulated enzyme. As can be seen in Figure 3B, IBMX superfusion stimulated cAMP production approximately 2-fold at 3 hrs and 4.5-fold at 24 hrs in the E7 transformed cells compared to the control cells, while the further cAMP elevation after forskolin (FSK) treatment was similar in both conditions. Altogether, these data suggest that, indeed, transformation of the cells by E7 stimulates adenylate cyclase-dependent production of cAMP above very low basal levels in the control cells. Figure 3C shows the relative increase in cAMP mobilization as pseudocolor changes in typical FRET experiments.

The article "HPV16 E7-Dependent Transformation Activates NHE1 through a PKA-RhoA-Iinduced Inhibition of p38alpha" was retracted in 2019. Reason: concerns about the images.

### Involvement of PKA and p38 in HPV16 E7-mediated transformation

To assess the role and dynamics of PKA and p38 in mediating transformation, we utilized changes in NHE1 activity as the transformation readout because we have previously demonstrated that stimulation of NHE1 occurs early in transformation and is necessary and sufficient for the further development of transformed phenotypes [48]. As seen in Figure 4, the induction of cellular E7 expression and transformation by removal of tetracycline for 24 hrs stimulated NHE1 activity by 69.5±6.2%, n = 15, P<0.02 (blue cross-hatched bar) and this stimulation was blocked by 2 µM of the specific inhibitor of the NHE1, HOE642 (data not shown). Inhibition of PKA by its specific inhibitor, H89, completely abrogated the transformation-dependent increase in NHE1 activity (green stippled bar) while inhibition of p38 activity by either its pharmacological inhibitor, SB203580, or by the transient expression of the dominant negative (dn) mutant for p38alpha (p38AF) further potentiated the transformation-dependent increase in NHE1 activity by approximately 2-fold (black stripped bars). Furthermore, inhibition of p38 either with SB203580 or via transient expression of dnp38alpha blocked the abrogation of the transformation-dependent activation of NHE1 by H89 (red stripped bars). These data strongly suggest that PKA and p38alpha are part of the same pathway in regulating the transformation-dependent stimulation of NHE1 and that PKA is up-stream of p38. This conclusion is further supported by the ability of H89 to block and forskolin (Fsk) to potentiate the E7-dependent down-regulation of p38 phosphorylation (Figures 4B & C) while having no effect on the phosphorylation state of JNK and ERK (Figure S4).

The article "HPV16 E7-Dependent Transformation Activates NHE1 through a PKA-RhoA-Iinduced Inhibition of p38alpha" was retracted in 2019. Reason: concerns about the images.

**Figure 4:** PKA is up-stream of p38 in regulating the HPV16 E7 expression-dependent stimulation of NHE1 activity. A. HPV16 E7 expression was induced by removing tetracycline from the culture medium for 24 hrs and the consequences on NHE1 activity of the specific inhibition for 24 hrs of PKA by 10^−7^ M of its specific inhibitor, H89, and/or p38 by either 10^−9^ M of its specific pharmacological inhibitor, SB203580, or by the transient expression of a dominant negative (dn) mutant for p38alpha (p38AF, 3 µg) was determined by spectrofluorometry using the pH sensitive probe BCECF-AM. Confluent monolayers were loaded with BCECF and placed in the perfusion cuvette and the monolayer perfused with 135 mM Na^+^ nominally bicarbonate free-HEPES ringer (pH 7.4) plus (Cont) or minus (E7) 2 µM tetracycline as previously described [48]. To analyze if PKA and p38 interact one each other in regulating NHE1 activity, cells were either first transfected with dnp38 for 48 hrs and then treated with H89 for 24 hrs or were simultaneosly treated with SB plus H89 for 24 hrs and NHE1 activity determined as above. Bars are mean±S.E. and the number of experiments ranged from 5 to 8. B. Non transformed (+tet) and transformed (−tet) cells were not treated (Cont) or treated with either 10^−7^ M H89 or 10−5 M FSK for 24 hrs and cells were homogenized as described in Materials and Methods. Aliquots containing 50 µg of protein were subjected to 10% SDS-PAGE and total and phosphorylated p38 was determined in Western Blot as in Figure 1. A representative immunoblot is shown. C. Summarized data of densitometrical analyses of p38 phosphorylation is represented as the relative ratio of the density of phospho-p38 against that of total p38. Relative ratio in control, non transformed cells was expressed as 1 arbitrary unit. Control cells are represented by dark bars, H89 treated cells by stippled bars and Fsk treated cells by cross-hatched bars. The data shown are mean values±S.E. (n = 4). p<0.05 (*) and p<0.01 (**) when compared with the control value by Student's t test.

### HPV16 E7-dependent transformation induces PKA-dependent phosphorylation and down-regulation of RhoA

However, the steps that mediate the down-regulation of p38 by PKA still need to be identified. RhoA is a potential candidate since it has been shown to be an upstream regulator of p38 in enhancing migration and invasion of breast cancer [11] and pancreatic carcinoma cells [32] and to be inhibited by PKA-dependent phosphorylation on serine 188 [11], [58]. If this is occurring during transformation then we would expect RhoA to be phosphorylated by PKA and to be inhibited by E7-dependent transformation. To test this hypothesis, we first measured the effect of transformation on the phosphorylation state of RhoA via Western Blotting analysis with antibodies specific for phosphorylated Ser-188 of RhoA (Fig. 5A) or via co-immunoprecipitation with anti-phosphoserine followed by anti-RhoA Western Blotting (Fig. 5B) at different times of HPV16 E7 expression (t0, 1 hr, 3 hr, 6 hr, 12 hr). Indeed, transformation induced a significant increase in RhoA phosphorylation in 2BN11 cells. A similar increase in RhoA phosphorylation was observed in E7 expressing HFK cells and late passage HPK1A cells (Figure S5) and blockage of NHE1 actvity with HOE642 had no effect on this process in either 2BN11 or HPK1A cells (Figure S3). To verify that this phosphorylation of RhoA observed upon transformation was due to PKA, we removed tet for 24 hrs in the absence or presence of a pharmacological PKA inhibitor (H89, 100 nM) or activator (forskolin, 10 µM) and we measured RhoA phosphorylation as above with the anti-phosphoSer188. The induction of phosphorylation was blocked by incubation with H89 and potentiated by incubation with forskolin (Fsk) during the time of induction of E7 expression (Fig. 5C).

The article "HPV16 E7-Dependent Transformation Activates NHE1 through a PKA-RhoA-Iinduced Inhibition of p38alpha" was retracted in 2019. Reason: concerns about the images.

**Figure 5:** HPV16 E7 induces PKA-dependent phosphorylation of RhoA. A. Western Blotting analysis of the phosphorylation state of RhoA at different times after tet removal (+tet, 1 hr, 3 hr, 6 hr and 24 hr) with antibodies specific for phosphorylated Ser-188 of RhoA (phospho RhoA) followed by polyclonal anti-RhoA antibody (total RhoA). B. Co-immunoprecipitation with anti-phosphoserine antibody followed by anti-RhoA Western Blotting (phospho RhoA) at different times of HPV16 E7 expression (t0, 1 hr, 3 hr, 6 hr, 24 hr). Expression of total RhoA in cell lysates was analyzed by immunoblot analysis using the polyclonal anti-RhoA antibody. C. To test if RhoA-phosphorylation induced by HPV16 E7 expression was dependent on PKA, tetracycline was removed and the cells either not treated or treated with either the pharmacological PKA inhibitor (H89, 100 nM) or activator (forskolin, 10 µM) and RhoA phosphorylation was measured as above (A).

As PKA can inhibit RhoA activity via its phosphorylation of serine 188, we next examined the effect of transformation on RhoA activity, first by a pulldown analysis of its binding to GST-fusion protein to the Rho binding domain of Rhotekin which associates preferentially with GTP-bound RhoA [59]. Figure 6A shows that the activity of RhoA was reduced upon E7-dependent transformation with a time course similar to that reported for the up-regulation of NHE1 activity by the same treatment [48] and for RhoA phosphorylation shown above and that H89 treatment blocked while forskolin (Fsk) treatment stimulated this reduction in RhoA activity. However, the biochemical detection of active RhoA via pull-down requires cell disruption and is performed in the presence of detergents which can lead to dissociation of preexisting complexes and, therefore, cause incorrect estimation of the extent of RhoA-GTP association to its down-stream effectors. In contrast, FRET microscopy permits the direct detection of the amount of active RhoA in intact living cells during E7-transformation. For this reason, we next measured RhoA activity state by using a a single-chain CFP/YFP FRET biosensor for RhoA (pRaichu 1297×) [60], which directly monitors the level of the endogenous RhoA-GTP by measuring FRET between the two pairs of GFP mutants fused to the Rho-Binding-Domain (RBD) of Rhotekin. Specifically, in this probe the binding of endogenous GTP-RhoA to RBD displaces YFP and CFP, thereby decreasing FRET efficiency. Using this FRET-based probe we verified that 24 hrs after tet removal, RhoA activity, which was assessed as the ratio of the CFP signal to the YFP signal, was significantly reduced (Figure 6B). Further, treatment with H89 during the transformation period completely reversed this E7-dependent inhibition of RhoA, again indicating that E7-induced RhoA inhibition was dependent on PKA.

The article "HPV16 E7-Dependent Transformation Activates NHE1 through a PKA-RhoA-Iinduced Inhibition of p38alpha" was retracted in 2019. Reason: concerns about the images.

**Figure 6:** HPV16 E7 expression activates NHE1 via a PKA-mediated-reduction in RhoA activity. A. Representative Western Blot of three GST-RBD pull-downs showing RhoA activity in 2BN11 cells at different times after tet removal and treated with 100 nM H89 and 10 µM FSK for the indicated times. The lower gel shows the amount of total RhoA in cell lysates. B. Sensitized FRET measurements of 2BN11 cells to determine the effect of E7 expression on RhoA activity in live cells. Cells were transfected with the RhoA biosensor pRaichu-1297× and then cultured with or without tet for 24 hr and treated or not with 100 nM H89 during the 24 hr period. Cells were imaged for CFP and FRET and the relative decreases in CFP/FRET ratios obtained (presented in the central column) indicate a decrease in active RhoA. Data are the mean±SEM from 32 to 37 different cells. ***P<0.005. CFP/FRET ratio images are in pseudocolor, with the color indicating the relative value at each pixel (lateral images), such that blue indicates the highest EmCFP/EmYFP ratio (highest RhoA activity), and red reflects the lowest EmCFP/EmYFP ratio (lowest RhoA activity). Scale bar is 10 µm. C. Role of PKA-mediated RhoA signalling on HPV16 E7-induced up-regulation of NHE1 activity. 2BN11 cells were transfected transiently with cDNA for either a phosphorylation dead (pd) RhoA mutant (blue cross-hatched bars), with dominant negative RhoA (dn) mutant (green stippled bars), with constitutively active RhoA (ca) (red striped bars) mutant or with siRNA against RhoA (brown reverse stippled bars). Control cells were transfected with the empty plasmid or non-specific siRNA transfected cells (scrambled) served as the control for RhoA silencing. After 24 hrs for cDNA construct or 48 hrs for siRNA transfection, tetracycline was then removed (−tet) or not (+tet) for a further 24 hrs and NHE1 activity was measured as described in Materials and Methods. Expression of these constructs had no effect on basal NHE1 activity in control, +tet cells. Inactivation of RhoA with the dn mutant and siRNA significantly potentiated the E7-induced stimulation of NHE1 activity while both activation of RhoA with the ca mutant and the block of RhoA phosphorylation by PKA with the pd mutant abrogated the E7-induced stimulation of NHE1 activity. Efficiency of siRNA-mediated RhoA knock-down was analyzed with immunofluorescence assay by using a monoclonal anti-RhoA antibody (green) and the blue fluorescent dye DAPI for staining nuclei (Figure S2).

The article "HPV16 E7-Dependent Transformation Activates NHE1 through a PKA-RhoA-Iinduced Inhibition of p38alpha" was retracted in 2019. Reason: concerns about the images.

In addition to phosphorylation by PKA, RhoA activity is controlled by the activity balance between other class of RhoA regulating proteins, the guanine nucleotide exchange factors (GEFs) and GTPase-activating proteins (GAPs) [29]. To assess if E7 alters the balance of GEFs and GAPs thus changing RhoA-GTP loading, we monitored the relative level of GEFs and GAPs in the presence and absence of tet for 24 hr, by using another FRET probe, pRaichu 1293×, consisting of a chimera of RhoA and the RhoA binding domain (RBD) of PKN, sandwiched between YFP and CFP. The relative increase in GEF activity increases the amount of GTP-RhoA and the intramolecular binding of GTP-RhoA to RBD and brings CFP in close proximity to YFP, resulting in an increase in FRET from CFP to YFP [60]. With this probe, we did not find any difference in the FRET ratio during E7-dependent transformation (0.8±0.031 vs 0.79±0.030, n = 20, n.s., for +tet and −tet, respectively) demonstrating that transformation did not influence GEF or GAP activity. These data suggest that a PKA-dependent phosphorylation of RhoA is the critical mechanism of E7 induced-RhoA inhibition.

### HPV16 E7 expression activates NHE1 through a reduction in RhoA activity via its phosphorylation on serine 188

While the preceding experiments indicate that RhoA is a substrate for PKA in these cells and that its phosphorylation at serine-188 is increased with E7-driven transformation, a critical question in the context of the current study is if the observed PKA-dependent phosphorylation and inhibition of RhoA is necessary for the transformation-dependent up-regulation of NHE1 activity. The phosphorylation of RhoA at serine 188 by PKA has been shown to block its action [46], [61], suggesting that this serine could be the PKA target also in our case. Therefore, as an approach to assess the role of PKA-dependent phosphorylation of RhoA in the activation of NHE1, we mutated the PKA phosphorylation site, serine188, to alanine to create a PKA phosphorylation dead (pd) RhoA mutant [11], [12]. Transfection of control 2BN11 cells with this pd RhoA^S188A^ mutant did not affect basal NHE1 activity levels of +tet cells, while it completely abrogated the increased NHE1 activity induced by expression of HPV16 E7 (Figure 6C, blue cross-hatched bars), confirming the requirement for PKA-dependent phosphorylation of RhoA at serine 188 for the up-regulation of NHE1 activity by E7-dependent transformation. We next determined if it is the alteration in RhoA activity utilizing either dominant negative (dn) mutants, constitutively active (ca) mutants [11] and/or expression utilizing an siRNA against RhoA that underlies stimulated NHE1 activity in transformed cells. Transient transfection of these constructs or the siRNA had no effect on NHE1 activity in +tet cells. Both inactivation of RhoA with the dn N19RhoA mutant (Figure 5C, green stippled bars) or the knock-down of its expression (Figure 6C, brown reverse stippled bars) significantly potentiated the E7-induced stimulation of NHE1 activity while activating RhoA with the ca V14RhoA mutant reduced this stimulation by approximately 80% (Figure 6C, red striped bars).

The article "HPV16 E7-Dependent Transformation Activates NHE1 through a PKA-RhoA-Iinduced Inhibition of p38alpha" was retracted in 2019. Reason: concerns about the images.

Altogether, these data demonstrate that the PKA-dependent phosphorylation of RhoA is a critical mechanism of HPV16 E7 induced-RhoA inhibition and it is an integral part of the PKA to p38alpha signal transduction module involved in the activation of the NHE1 during transformation.

## Discussion

There still is a dearth of data concerning the very early signal transduction events regulating neoplastic transformation- the first step of the carcinogenic process that is limited to the altered cell. The elucidation of the underlying alterations in signal transduction events mediating the initiation, development and regulation of transformation is a necessary prerequiste for understanding the origin and early development of cancer. As discussed in [17], to accomplish this it is necessary to use an experimental model in which the transformation of a normal, immortalized cell by a single oncogene can be highly controlled, thus permitting the dissection of the sequence of events occuring after the initial alteration and the role of a particular gene or signal transduction pathway. These cells, unlike cancer-derived cell lines, have not aquired genomic instability nor unspecific genetic and epigenetic alterations that can mask the specific transformation-dependent alterations.

We utilized this type of inducible cell model with the E7 oncogene of HPV16 to dissect the sequence of the very early steps in signal transduction underlying “the moment” in which a still normal cell becomes transformed. To accomplish this, NIH-3T3 cells were transfected with a construct in which E7 gene expression is under the control of a promoter that is negatively regulated by tetracycline so that E7 is expressed only after tetracycline removal [48] (clone 2BN11). Using this model system, we previously reported that the development of transformed phenotypes (*e. g.* increased proliferative rate, anchorage-independent growth, serum independence and increased glycolytic metabolism) are under the strict control of E7 expression in these cells and, further, that intracellular alkalinization driven by an up-regulation of the Na^+^/H^+^-exchanger (NHE1) is a very early physiological event in transformation and which, in turn, is necessary for the development and maintenance of many of the cellular events occurring later in the transformation process such as serum independence, increased growth rate, anchorage-independent growth and *in vivo* tumour development in nude mice. For this reason, we here utilized changes in NHE1 activity as the readout for the analysis of the role of a particular signal transduction pathway in transformation in the dissection of the early signaling events occurring up-stream of NHE1 activation during E7-dependent transformation.

This experimental model enabled us to recognise and follow a strictly defined sequential progression arising from the initial expression of E7 that rapidly transforms the cells. Our data demonstrate that an intracellular mobilization of cAMP is one of the first signaling events occurring during transformation (Figure 3). Further, we provide evidence that this initial rise in cAMP is followed by a PKA-dependent inhibition of RhoA activity (Figures 6A and 6B) which is necessary for the inactivation of p38alpha (Figure 4B) and which, in turn, regulates the subsequent E7-mediated transformation–dependent early stimulation of NHE1 activity (Figures 4A and 6C). Although the individual importance of each of these signal systems in tumor induction both *in vitro* and *in vivo* is well documented, their interrelations in mediating transformation were heretofore still unknown.

The article "HPV16 E7-Dependent Transformation Activates NHE1 through a PKA-RhoA-Iinduced Inhibition of p38alpha" was retracted in 2019. Reason: concerns about the images.

Indeed, while there is now much data demonstrating the tumor suppressor role of p38 MAP Kinase (see introduction), to date it has not been demonstrated whether the down-regulation of p38alpha plays a role in the early induction of cellular events leading to transformation. Further, if it is involved in transformation, we asked at which point is it located in the transformation process, which up-stream mechanisms regulate its inhibition and what is its down-stream target. We first demonstrated in NIH3T3 cells and in human primary (HPK1A) and secondary (HFK) keratinocytes that E7-dependent transformation specifically reduces p38 phosphorylation. Then, using the inducible experimental model we show that p38alpha plays a key role in the acquisition of the increased activity of the NHE1 which sets the stage for the development of the other transformed phenotypes [48]. Interestingly, p38alpha has also been found to have a negative role in regulating both migration and invasion of pancreatic and breast carcinoma cells [11]–[12], [32] and its activity is reduced in hepatocellular carcinomas in comparison to adjacent normal tissue [62], suggesting that its down-regulation is not limited to just transformation and early tumorigenesis but also in later metastatic/aggressive stages.

The involvement of the cAMP/PKA pathway in mediating tumor progression [35] together with the demonstrated integration of p38 with cAMP/PKA signaling in different cell systems [43], [57], [63], [64] focused our attention on the possibility that E7 transformation-dependent down-regulation of p38 involves the cAMP/PKA system. Transformation induced substantial increase in adenylate cyclase-dependent cellular cAMP mobilization (Fig. 2) and incubation with the PKA selective inhibitor, H89, during E7-dependent transformation blocked the down-regulation of p38 phosphorylation while stimulation of the cAMP/PKA system by forskolin (Fsk) enhanced this E7-dependent down-regulation of p38 phosphorylation (Fig. 4B and 4C). Further, inhibition of p38 with either SB203580 or via transient expression of a dominant negative p38alpha mutant (dn p38alpha) blocked the H89-dependent abrogation of the transformation-dependent activation of NHE1 (Figure 3A), further supporting the suggestion that PKA and p38alpha belong both physically and functionally to a common signalling unit, in which PKA acts up-stream to p38 in regulating the transformation-dependent stimulation of NHE1 activity.

As RhoA is known be a PKA-signalling effector in a plethora of cell responses [11], [58], [44] and to play an important role in regulating p38 kinase activity in several cellular regulatory contexts [11], [32], [63], [64], we analysed its involvement in underlying the down-regulation of p38 by PKA and in their regulation of E7-dependent activation of NHE1. We observed that RhoA was rapidly phosphorylated at Ser-188 upon E7 expression (Figs. 4A & B) and PKA is involved in this phosphorylation since inhibition of the kinase with H89 or its stimulation by forskolin (Fsk) during the time of induction of E7 expression respectively blocked or potentiated the E7-induced phosphorylation (Fig. 4C). Further, RhoA was inhibited upon E7 expression with a time course parallel to its E7-induced phosphorylation (Figures 6A & B) and inhibition of PKA by H89 reversed the decrease in RhoA activity only in transformed cells (Figure 6B). Interestingly, FRET measurements of Rho-GEFs/GAP activity revealed that the inhibition of RhoA via changes in their activity could be excluded during E7 transformation. Altogether these data suggest that the PKA that is activated in HPV16 E7 transformed cells inhibits RhoA activity through its phosphorylation of RhoA at serine 188. RhoA has been recently reported to be inhibited as a result of transformation driven by TGFbeta [67] or, importantly, HPV16 E7 expression [33] suggesting that this might be a common mechanism. An important question was if the observed PKA-dependent phosphorylation and inhibition of RhoA is necessary for the transformation-dependent up-regulation of NHE1 activity. Analysis of NHE1 activity after transfection of a dn RhoA mutant or siRNA to block RhoA function/expression or a ca RhoA mutant to enhance RhoA function (Figure 6C) demonstrated the importance of the inhibition of RhoA activity in E7 transformation-induced NHE1 activity while transfection of the phosphodead (pd) RhoA mutant revealed the important role for its PKA-dependent phosphorylation in E7 transformation-induced NHE1 activity.

The article "HPV16 E7-Dependent Transformation Activates NHE1 through a PKA-RhoA-Iinduced Inhibition of p38alpha" was retracted in 2019. Reason: concerns about the images.

The activity of many enzymes is strictly controlled by intracellular pH (pHi) and, therefore, an important question is what extent this E7-induced signal cascade described herein might be altered via feedback by the changes in pHi driven by the stimulated NHE1 [48]. To address this question, we measured cAMP production, phosphorylation of RhoA and the inhibition of p38 in the presence and absence of 2 µM HOE642, a potent and specific inhibitor of the NHE1, in both 2BN11 cells and in early and late passages of HPK1A cells. This treatment has been previously shown to block the development of phenotypes down-stream of the NHE1 in both cell lines [48]. As can be seen in Figure S3, this treatment had no effect on any of these process in either of the cell lines suggesting a strict unidirectionality of this signal cascade both in the rat fibroblast and human keratinocyte models.

In conclusion, in this study we have recognised a strictly defined sequential progression arising from the initial expression of E7 that rapidly transforms the cells. Our data demonstrate that an intracellular mobilization of cAMP is one of the first signaling events occurring during transformation and that this initial rise in cAMP is followed by a PKA-dependent inhibition of RhoA activity which is necessary for the inactivation of p38alpha which, in turn, regulates the subsequent E7-mediated transformation–dependent early stimulation of NHE1 activity. An important question is whether this signal cascade is engaged by simple E7 expression or is transformation dependent. The data in Figure 1D shows that only transformation competent E7 is able to inhibit p38 and the use of the HPK1A model system in this study, in which the original viral infection (early passage) simply immortalizes the cells and with time they become transformed (late passage), further validated the concept of transformation specific effects. Importantly, finding the same signal transduction cascade turned on in the late passage HPK1A cells also demonstrated that this signal cascade is engaged during the natural progression of primary human keratinocyte cells that were infected with the actual HPV16 virus and is not just a consequence of the expression of a single viral gene as was also observed previously for NHE1 activity [48]. The elucidation of these signal transduction systems and, more importantly, their interrelations in the early stages of the HPV-dependent transformation processes could provide indications for novel therapeutic strategies and/or a potential marker test for the clinical determination of pre-cancer, HPV-transformed cells in the cervix.

## Supporting Information

Figure S1 Effect of pharmacological treatment and transfection of cDNA plasmids on E7 message expression by RT-PCR analysis. 2BN11 cells were treated with each of the pharmacological agents or transfected with the indicated cDNA encoding vectors as described in Results. RNA was extracted and 500 ng of each sample total RNA were subjected to a semi-quantitative RT-PCR for HPV16 E7 expression analysis. GAPDH: loading control.
(0.07 MB TIF)

Figure S2 Analysis by immunofluorescence microscopy of the decrease in RhoA expression by RNAi in 2BN11 cells. A. Cells were transfected with either control, non-targeting siRNA (left panel) or RhoA specific siRNA (right panel) as described in Materials and Methods. RhoA was visualized with Alexa Fluor 488 (green) and the nuclei with DAPI (blue). B. Quantification of the intensity of RhoA signals through the cell area normalized to cell number. Data represent mean±SE of three independent experiments.
(1.35 MB TIF)

Figure S3 Monolayers of either 2BN11 or HPK1A were treated or not with 2 µM of the specific NHE1 inhibitor, HOE642, and analyzed for cAMP, phospho-RhoA or phospho-p38 levels as described in Materials and Methods. In 2BN11 cells the measurements were made in the presence of tetracycline (+tet) or 3 or 24 hours after its removal while in HPK1A cells the comparison was between early and late passage cells.
(0.21 MB TIF)

Figure S4 Non transformed (+tet) and transformed (−tet) cells were not treated (Cont) or treated with either 10−7 M H89 or 10−5 M FSK for 24 hrs and cells were homogenized as described in Materials and Methods. Aliquots containing 50 µg of protein were subjected to 10% SDS-PAGE and total and phosphorylated JNK (upper blot) or ERK1/2 (lower blot) was determined in Western Blot as in Figure 1. A representative immunoblot is shown for each MAP kinase.
(0.39 MB TIF)

Figure S5 Western Blotting analysis of the phosphorylation state of RhoA in HFK or HPK1A cells with antibodies specific for phosphorylated Ser-188 of RhoA (phospho RhoA) followed by polyclonal anti-RhoA antibody (total RhoA). A representative immunoblot is shown for each. HFK cells were infected with empty pLXSN vector or pLXSN vector containing wild-type, non-tagged E7 while HPK1A early passage cells were compared with late passage cells.
(0.13 MB DOC)
